# Timing of Acupuncture Treatment in Peripheral Facial Paralysis: A Systematic Review and Meta-Analysis

This article has been retracted.

**DOI:** 10.1155/2021/4221955

**Published:** 2021-12-15

**Authors:** Zelin Yu, Mengxia Shen, Wenfang Shang, Jiangxia Wu, Lihua Xuan

**Affiliations:** ^1^The First Clinical Medicine College, Zhejiang Chinese Medical University, Hangzhou, Zhejiang 310053, China; ^2^The First Affiliated Hospital of Zhejiang Chinese Medical University, Hangzhou, Zhejiang 310006, China

## Abstract

**Objective:**

Investigate the optimum time of acupuncture treatment in peripheral facial paralysis in order to provide evidence for clinical treatment.

**Methods:**

CNKI, Wanfang, PubMed, Cochrane Library, and EMBASE databases were systematically searched from the inception dates to February 20, 2020. Studies limited to participants with acute peripheral facial paralysis treated with acupuncture and patients without information of the stage were excluded. The primary outcomes were effective rate and cure rate (based on facial nerve function scores). This meta-analysis is registered with PROSPERO, number CRD42020169870.

**Results:**

15 randomized controlled trials that enrolled 2847 participants met the selection criteria. There was no significant differences in the effective rate (RR, 1.22; 95% CI, 0.70-2.11) when comparing acupuncture to prednisone therapy in acute facial paralysis. Acupuncture treatment in the acute stage increased both the effective rate (RR, 1.03; 95% CI, 1.00-1.07) and the cure rate (RR, 1.34; 95% CI, 1.14-1.58) compared to that in the nonacute stage.

**Conclusions:**

In this meta-analysis, acupuncture showed a better effect in the acute stage than the nonacute stage for participants with peripheral facial paralysis. There was no statistical difference in the effective rate no matter the choice of acupuncture or prednisone therapies in the acute stage. These findings encourage early acupuncture treatment in peripheral facial paralysis.

## 1. Introduction

Peripheral facial paralysis is an acute facial palsy due to the inflammation of the facial nerve [1]. It is a kind of self-limited disease, and its clinical manifestation is distortion of the face as well as interference with nerve functions [2]. Hitherto, its definite etiology is still inexplicit. According to the data from Morris et al., there are more than 60,000 people who developed Bell's palsy in the United States per year [3], while epidemiological investigation shows that about 420,000 people get facial palsy in China [4]. Hence, the treatment of facial paralysis has collected extensive attention over the world. According to the guideline, early oral antiviral therapy in addition to oral steroids is strongly recommended. But after steroid treatment, there is no other way except B vitamins and alternative therapies such as acupuncture [5]. Although Bell's palsy is self-limited, there are still over 10% of patients who cannot get complete recovery and get long-term sequelae. Hence, it is necessary to find an optimal therapeutic schedule.

In China, there has been a long history of acupuncture in the treatment of peripheral facial paralysis, where it is called “deviated mouth.” According to the report of WHO in 1979, peripheral facial paralysis is one of the dominant diseases of acupuncture [6]. However, there has been longstanding controversy about when acupuncture should be given [7]. The course of peripheral facial paralysis is divided into three stages: acute stage (1~7 days), quiescent stage (8~14 days), and recovery stage (over 15 days) due to the inflammatory edema and emergence of sequelae. Mengyuan et al. [8, 9] performed a study and claimed that in the acute stage (in 7 days), acupuncture stimulation may aggravate the edema of nerve tissue, increase the pressure of the facial nerve canal, and accelerate the degeneration of the facial nerve. Dage and Boldbayar [10] found out that there was a refractory period (no response to treatment including acupuncture) at the early age of peripheral facial paralysis. However, as the evidence began to accumulate, more trials suggested that patients recovered better with early acupuncture intervention.

Thus, the primary objective of our study was to systematically review randomized controlled trials investigating timing of acupuncture treatment in peripheral facial paralysis.

## 2. Methods

### 2.1. Search Strategy

For this meta-analysis, we searched the CNKI, Wanfang, PubMed, Cochrane Library, and EMBASE databases from inception to Feb. 20, 2020, without language restrictions, for randomized controlled trials that compared the use of acupuncture in the acute stage with the nonacute stage of peripheral facial paralysis. Full search terms and search strategy are provided in Table 1.

### 2.2. Selection Criteria

Trials were included for the following inclusion criteria: (1) those with patients who were treated for peripheral facial paralysis, (2) randomized controlled trials, and (3) comparisons of acupuncture and placebo or drug therapy in the acute stage or comparisons of acupuncture treatment in the acute stage and nonacute stage.

Exclusion criteria were (1) those without a clear definition of the acute stage (the number of days of onset), (2) randomized trials without a control group, (3) trials in which acupuncture was combined with other treatments (e.g., Chinese herbs), and (4) studies of comparison of 2 different acupuncture methods.

### 2.3. Risk-of-Bias Assessments

The methodological quality of the included RCTs was assessed by two authors (Yu and Shang) independently based on Cochrane risk-of-bias criteria. Each quality item was graded as low risk, high risk, or unclear risk. The 7 items used to evaluate bias in each trial included the randomization sequence generation, allocation concealment, blinding of participants and personnel, blinding of outcome assessment, incomplete outcome data, selective reporting, and other biases [11].

We defined other biases as trials in which baseline characteristics were not similar between different intervention groups. Publication bias was assessed using funnel plots.

### 2.4. Data Extraction

Two reviewers (Yu and Shang) extracted data independently, and in duplicate, extracted the following information from each study: author, publication year, acupoint selection, acupuncture methods, country of origin, drugs, trial duration, and participant characteristics. When it came to a disagreement, Wu would make the final judgement. If the trials had more than 2 groups or factorial designs and permitted multiple comparisons, we extracted the data of interest in the original articles.

The primary outcome was cure rate and effective rate.

### 2.5. Data Analysis

The association of acupuncture, drugs, and combined acupuncture and drugs with efficacy and cure rate was assessed, and whether the therapy was taken in the acute stage or not was compared. We performed meta-analysis to calculate risk ratios (RRs) with 95% CIs using the Mantel-Haenszel statistical method. Based on the practice recommendation of the Cochrane Handbook [8], trials with zero events in both the intervention and control groups were not included in the meta-analysis when RRs were calculated.

Statistical heterogeneity between summary data was evaluated using the *I*^2^ statistic. Then, we decide whether a random-effects model or a fixed-effects model was to be used to pool the data. Sensitivity analysis was performed by excluding low-quality studies.

Prespecified subgroup analyses for the main outcome included published year (before 2013 vs. after 2013), sample sizes (<150 vs. ≥150), intervention method (acupuncture vs. acupuncture combined with drugs), and acupoint selection. (principle point vs. principle point+supplementary points based on different symptoms vs. supplementary points based on different syndromes).

The sensitivity analysis was analyzed using Stata 14.0 (Stata Corporation, College Station, TX), and the rest of the available data were analyzed using RevMan 5.3 (The Nordic Cochrane Centre, Copenhagen, Denmark).

## 3. Result

### 3.1. Studies Retrieved and Characteristics

Our search identified 1385 potentially eligible records. And once duplicates had been removed, 696 records were screened, of which 98 full texts were assessed for eligibility. Finally, 15 texts [12–26] involving 2847 participants met the inclusion criteria.  Figure 1 outlines the search process.

Table 2 shows the characteristics of the 15 included trials. All the included RCTs were published from 2004 to 2020, and all were performed in China. All the studies reported acupoint selection and manipulation while 5 trials [13, 17, 19, 21, 22] failed to report the size of the needle. A range of outcome measures were used individually and in combination to evaluate the benefits of acupuncture for peripheral facial paralysis across studies in relation to nerve function, quality of life, psychological condition, blood index, and electrophysiology. 14 studies calculated effective rate, and 10 studies calculated the cure rate according to the curative effect standard [27, 28]. The definition of the different levels of curative effect was based on facial nerve function scores [27–30]. Two studies reported side-effects.

Included studies were assessed using the Cochrane Collaboration's Risk of Bias tool [11] (Figure 2). All studies are randomized. Because of the characteristic of acupuncture therapy, it is difficult to achieve double-blind. Studies usually adopted the single-blind method, and participants did not know which group they would be assigned to. 15 trials described an adequate random sequence generation process, 4 trials described the methods used for allocation concealment, and all studies had an unclear risk of other biases. 11 trials were of low quality while 4 of high quality.

We deleted one single study from the overall pooled analysis each time to check the influence of the removed data set to the overall RRs. After the deletion of the study by Wu et al., the heterogeneity decreased significantly, while the association still kept significant. We found out that Wu et al. observed outcomes after 6 months rather than one or two months like other trials. A sensitivity analysis by Stata was performed, and the trial was excluded (Figure 3).

### 3.2. Efficacy of Acupuncture Compared with Drugs

Five studies which included 595 individuals compared acupuncture therapy with drugs. As is shown in Figure 4, there was no statistically significant association of the intervention with the effective rate (RR, 1.22; 95% CI, 0.70-2.11; *I*^2^ = 98%, *P* < 0.00001) and the markedly effective rate (RR, 1.53; 95% CI, 0.98-2.86; *I*^2^ = 89%, *P* < 0.00001). Acupuncture therapy was associated with an increased cure rate (RR, 1.66; 95% CI, 1.27-2.19, *I*^2^ = 0%, *P* = 0.61).

### 3.3. Efficacy of Acupuncture Treatment at Different Stages

Seven trials which included 1786 individuals compared the acute treatment with the nonacute treatment. The acute acupuncture treatment was associated with an increased effective rate (RR, 1.03; 95% CI, 1.00-1.07, *I*^2^ = 0%, *P* = 0.57) as well as an increased cure rate (RR, 1.34; 95% CI, 1.14-1.58), with moderate heterogeneity in the pooled results (*I*^2^ = 61%, *P* = 0.02). The L'Abbe graph and the Galbraith plot shown in Figures 5 and 6, respectively, also suggest certain heterogeneity, which means subgroup analysis is imperative.

Table 3 summarizes results of subgroup analyses for acupuncture treatment in different stages. It is worth mentioning that we noticed that in some studies [13, 18, 23, 26], acupuncture treatment was given after the acute stage in the control group and ended at the same day as the experimental group. In other words, although drug treatment lasted for a consistent time in both groups, acupuncture time in the experimental group was 7 days longer. So besides prespecified subgroups, we added another subgroup of acupuncture time. The subgroup analysis showed similar results across subgroups based on published year, intervention method, and acupoint selection.

Visual inspection of funnel plots (Figures 7 and 8) suggested there was no extreme publication bias for both the cure rate and the effective rate.

## 4. Discussion

Results of this meta-analysis provide strong evidence that acupuncture in the acute stage of peripheral facial paralysis benefits the patients. Acute acupuncture treatment was associated with an increased effective rate and cure rate. Sensitivity analyses that excluded low-quality trials did not alter these results. Moreover, these results were generally consistent regardless of the published year, intervention method, and acupoint selection. There are some theories about the physiologic mechanism of acupuncture treatment, including anti-inflammation and enhancing blood circulation. Li et al. [31] proved that acupuncture can activate CRH neurons in the paraventricular nucleus and increase plasma ACTH level in order to reduce inflammation. Lim et al. [32] found out acupuncture can decrease the level of proinflammatory factors through the cholinergic anti-inflammatory pathway so as to play a rapid, direct, and effective anti-inflammatory effect. Li et al. [33] suggested that acupuncture can increase skin microcirculation blood perfusion.

The subgroup analyses of sample sizes and acupuncture time happened to have the same grouping. And the results showed a decrease of heterogeneity and significant differences between subgroups. Since we admitted the efficacy of acupuncture, four trials [13, 18, 23, 26] showed longer treatment times, which might have increased the probability of bigger RRs of the experimental group. These trials exaggerated the efficacy of acupuncture treatment. The large sample group may have a more rigorous study design and avoided the variation of acupuncture time, which is reasonable.

This study has several limitations. First, because of the characteristic of acupuncture therapy, it is difficult to achieve double blind. Thus, the placebo effect is difficult to rule out. Second, the outcome index of the included studies was not enough. Third, the standard of effectivity and cure was not the same exactly for all studies. Fourth, all the trials were from China which hindered the applicability exploration of acupuncture in more regions and ethnic lines. Fifth, records of side-effect or accidents during the acupuncture treatment were not mentioned in most studies, so that the safety cannot be evaluated.

## 5. Conclusions

Acupuncture, from the present trials, showed a better effect in the acute stage than the nonacute stage for participants with peripheral facial paralysis. There was no statistical difference in the effective rate no matter the choice of acupuncture or prednisone therapies in the acute stage. These findings encourage early acupuncture treatment in peripheral facial paralysis. More high-quality RCTs from all regions are needed. Please carefully refer to the conclusions of this meta-analysis.

## Figures and Tables

**Figure 1:** Study selection.

**Figure 2:** Risk of bias ratings.

**Figure 3:** Sensitivity analysis.

**Figure 4:** Meta-analysis results of acupuncture compared with drugs for acute peripheral facial paralysis.

**Figure 5:** L'Abbe graph.

**Figure 6:** Galbraith plot.

**Figure 7:** Funnel plot of effective rate.

**Figure 8:** Funnel plot of cure rate.

**Table 1:** Search strategy for each database.

Database	Search strategy
PubMed	#1 “acupuncture” [MeSH terms] OR “acupuncture” [all fields] #2 “electroacupuncture” [MeSH terms] OR “moxibustion” [all fields] OR “moxibustion” [MeSH terms] #3 “peripheral facial paralysis” [MeSH terms] OR “peripheral facial paralysis” [all fields] #4 “paralyses, facial” [all fields] OR “paralysis, facial” [all fields] OR “facial palsy” [all fields] OR “facial palsies” [all fields] OR “facial palsy, lower motor neuron” [all fields] OR “lower motor neuron facial palsy” [all fields] #5 “acute phase” [all fields] OR “acute” [all fields] #6 #1 or #2 #7 #3 or #4 #8 #5 and #6 and #7

EMBASE	#1. “acupuncture”/exp OR “acupuncture” OR “moxibustion”/exp OR “moxibustion” #2. “peripheral facial paralysis” OR “lower motor neuron facial palsy” OR “bell palsy” #3. “acute” OR “acute stage” OR “acute phase” #4. #1 AND #2 AND #3

Cochrane Library	#1 acupuncture (word variations have been searched) #2 moxibustion (word variations have been searched) #3 peripheral facial paralysis (word variations have been searched) #4 lower motor neuron facial palsy (word variations have been searched) #5 acute phase (word variations have been searched) #6 acute stage (word variations have been searched) #7 #1 OR #2 #8 #3 OR #4 #9 #5 OR #6 #10 #7 AND #8 #11 #10 AND #9

Wanfang	#1 acupuncture or acupuncture therapy #2 peripheral facial paralysis or Bell's facial paralysis #3 acute or early

CNKI	#1 acupuncture or acupuncture therapy #2 peripheral facial paralysis or Bell's facial paralysis #3 acute or early

**Table 2:** Characteristics of included trials and participants.

Included trials	Intervention			Participants			Treatment duration
	Acute stage	Quiescent recovery stage	Recovery stage	Sample size, *n*	Mean age, years ± SD	Men, *N* (%)	
Liang 2004	ACU; ACU+D; D	ACU; ACU+D		480	40.1 ± 15.1	249 (51.9%)	30 d
Wu 2006	ACU+D	ACU+D		150	41.0 ± 17.2	71 (47.3%)	60 d
Shen 2009		ACU+D		279	46.7 ± 31.3	141 (50.5%)	60 d
Qin 2013	ACU+D	ACU+D	ACU+D	120	43.1 ± 15.2	57 (50.9%)	30 d
Chen 2018	ACU; D			86	47.6 ± 3.4	47 (54.7%)	10 d
Yang2018	ACU; D			84	47.2 ± 2.8	51 (60.7%)	36 d
Dong2018	ACU; D			70	40.5 ± 5.0	44 (62.9%)	28 d
Mao 2019	ACU; ACU+D		ACU+D	90	42.2 ± 16.7	43 (47.8%)	30 d
Wang 2019	ACU	ACU+D		100	42.0 ± 1.3	57 (57.0%)	30 d
Zhou 2019	ACU+D	ACU+D		60	41.7 ± 12.5	34 (56.7%)	30 d
Song 2019	ACU	ACU		62	45.0 ± 5.2	37 (59.7%)	
Li 2011	ACU	ACU	ACU	891	40.5 ± 15.4	469 (52.6%)	28 d
Yang 2014	ACU; D			120	41.7 ± 10.6	70 (58.3%)	28 d
Liu 2017	ACU; D			84	46.5 ± 16.2	40 (47.6%)	28 d
Wang 2018	ACU+D	ACU+D		134	37.7 ± 12.7	63 (47.0%)	28 d

**Table 3:** Subgroup analysis of acupuncture for peripheral facial paralysis in acute stage or nonacute stage.

Variable	No. of trials	No. of participants		Cure rate, RR (95%)	Heterogeneity	Subgroup differences
		Cured	Total			
Published year						
≤2013	4	766	1532	1.26 [1.06, 1.50]	*P* = 0.04; *I*^2^ = 64%	0.28
>2013	3	142	254	1.61 [1.08, 2.40]	*P* = 0.18; *I*^2^ = 42%	
Intervention^∗^						
ACU	2	484	1047	1.17 [0.96, 1.43]	*P* = 0.18; *I*^2^ = 42%	0.18
ACU+drugs	6	424	739	1.49 [1.12, 1.98]	*P* = 0.18; *I*^2^ = 42%	
Sample size						
<150	4	190	366	1.71 [1.25, 2.35]	*P* = 0.14; *I*^2^ = 46%	0.02
≥150	3	718	1420	1.15 [1.06, 1.25]	*P* = 0.64; *I*^2^ = 0%	
Acupoint						
Acupoint^1^	2	298	529	1.20 [0.94, 1.54]	*P* = 0.004; *I*^2^ = 82%	0.48
Acupoint^2^	3	493	1063	1.69 [0.99, 2.87]	*P* = 0.56; *I*^2^ = 0%	
Acupoint^3^	2	117	194	1.36 [1.08, 1.71]	*P* = 0.02; *I*^2^ = 61%	
ACU time						
Same	3	718	1420	1.15 [1.06, 1.25]	*P* = 0.64; *I*^2^ = 0%	0.02
Vary	4	190	366	1.71 [1.25, 2.35]	*P* = 0.14; *I*^2^ = 46%	

Note: Acupoint^1^: principle point; Acupoint^2^: principle point+supplementary points based on different symptoms; Acupoint^3^: principle point+supplementary points based on different syndromes. ^∗^ Fangrong et al. [12] studied both acupuncture and acupuncture in addition to drug in different stages. So this study was counted in two groups and added up to 8.

## Data Availability

The data used to support the findings of this study are available from the corresponding author upon request.
